# Modeling and Analysis of Breast Cancer with Adverse Reactions of Chemotherapy Treatment through Fractional Derivative

**DOI:** 10.1155/2022/5636844

**Published:** 2022-02-12

**Authors:** Tao-Qian Tang, Zahir Shah, Ebenezer Bonyah, Rashid Jan, Meshal Shutaywi, Nasser Alreshidi

**Affiliations:** ^1^International Intercollegiate Ph.D. Program, National Tsing Hua University, Hsinchu 30013, Taiwan; ^2^Department of Internal Medicine, E-Da Hospital, Kaohsiung 82445, Taiwan; ^3^School of Medicine, College of Medicine, I-Shou University, Kaohsiung 82445, Taiwan; ^4^Department of Family and Community Medicine, E-Da Hospital, Kaohsiung 82445, Taiwan; ^5^Department of Engineering and System Science, National Tsing Hua University, Hsinchu 30013, Taiwan; ^6^Department of Mathematical Sciences, University of Lakki Marwat, Lakki Marwat, 28420 KPK, Pakistan; ^7^Department of Mathematics Education, University of Education Winneba Kumasi (Kumasicompus), Kumasi 00233, Ghana; ^8^Department of Mathematics, University of Swabi, Swabi, 23561 KPK, Pakistan; ^9^King Abdulaziz University, College of Science & Arts, Department of Mathematics, Rabigh, Saudi Arabia; ^10^Department of Mathematics College of Science Northern Border University, Arar 73222, Saudi Arabia

## Abstract

The abnormal growth of cells in the breast is called malignancy or breast cancer; it is a life-threatening and dangerous cancer in women around the world. In the treatment of cancer, the doctors apply different techniques to stop cancer cell development, remove cancer cells through surgery, or kill cancer cells. In chemotherapy treatment, powerful drugs are used to kill abnormal cells; however, it has adverse reactions on the patient heart which is called cardiotoxicity. In this paper, we formulate the dynamics of cancer in the breast with adverse reactions of chemotherapy treatment on the heart of a patient in the fractional framework to visualize its dynamical behaviour. We listed the fundamental results of the fractional calculus for the analysis of our model. The model is then analyzed for the basic properties, and the existence and uniqueness of the proposed breast cancer system are investigated through fixed point theory. Furthermore, the Adams-Bashforth numerical technique is presented for the solution of fractional-order system to illustrate the time series of breast cancer model. The dynamical behaviour of different stages of breast cancer is then highlighted numerically to show the effect of fractional-order *ϑ* and to visualize the role of input parameter on the dynamics of breast cancer.

## 1. Introduction

Medical experts reported that breast cancer is the abnormal growth of cells in the breast which is a life-threatening disease and is mostly found in women. It is reported in [1] that breast cancer has the highest incidence rate as compared to the other cancer types. It destroys breast tissue and breast cells to grow out of control and to change the breast to abnormal shape. After lung cancer, breast cancer is declared to be the largest cancer in the globe, and every woman may be infected by this infection. It is stated by the WHO that about 8 to 9 percent of the women are infected by breast cancer in the world; moreover, the root cause is not yet explored by the medical experts. However, several risk factors are predicted which increase the risk of breast cancer in women which include dietary arrangements, drinking alcohol, smoking, being a woman, dense breast, lack of exercise, pregnancy history, genetic, breastfeeding history, race, menstrual history, life history, weight, certain breast changes, personal history of breast cancer, and age. The main symptoms of breast cancer are swollen lymph node nipple discharge, pulling in of the nipple, breast or nipple pain, flaky skin on the breast or nipple, irritation of the skin, dimpled skin red, a change in the size or shape of a breast, thickening of part of a breast, and full or partial swelling.  Figure 1 is the representation of breast or milk making factory for the newly baby child with cancer cells which further grow and damage the body of infected individuals.

Medical authorities assess cancer condition of a patient by using stages, and these stages are tumor, node, and metastasis which determine the chances of recovery from cancer. The early the stage, the greater the chances of recovery. Numerous treatment techniques have been developed for prevention of cancer which includes surgery, gene therapy, bisphosphonates, immunotherapy, targeted cancer drugs, hormone therapy, bone marrow transplants and stem cell, cancer drugs, radiotherapy, and complementary and alternative therapies. The most common treatment of the above is chemotherapy which involves the use of drugs to kill cancer cells. In chemotherapy, the drugs are either injected to the patient or are used orally which have some effectiveness but may hurt the heart. This bad side effect is called cardiotoxicity and affects children and adults [2]. The failure of patient heart is reported and observed during oncological treatment of anthracyclines and trastuzumab [3]. It is still a challenge for cancer expert and cardiologists to prevent cardiotoxicity experience during chemotherapy treatment. In chemotherapy treatment, anthracycline drugs are used which affect the heart of the patient and lead to cardiotoxicity illustrated in Figure 2.

Mathematical frameworks are used to conceptualize the intricate dynamics of diseases and to provide accurate results for the control and prevention of these infections [4, 5]. In modeling of cancer, the journey starts from 1954 [6] to explain cancer, and then, the researcher studies different aspects of cancer and tumor growth [7, 8]. A mathematical model of chemotherapy treatment for cancer has been developed by Dixit et al. [9]; the authors represent the treatment procedure for tumor cancer. The dynamics of cancer represent the interactions of tumor cell energy and tumor cell density and the effect of chemotherapy drugs. Recently, a mathematical model has been formulated for low-dose chemotherapy with minimal parameters; they studied angiogenic signals between vasculature and tumors [10]. In [11], a compartmental model has been developed by Jordao and Tavares; they consider cancerous and healthy cells to analyze the proposed model of cancer. The role of time delay on the dynamic of tumor system has been investigated by S. Khajanchi and Nieto [12]. Another important model was developed by Mahlbacher et al. [13] to conceptualize the interactions between immune and tumor and predict better suggestions about cancer. In the literature, several mathematical models have been developed and formulated to study, conceptualize, and visualize the transmission phenomena of cancer [14–17].

Recent advancement of fractional calculus showed that the results of fractional operators are more accurate, precious, and reliable as compared to the system of classical derivatives [18, 19]. Novel fractional operators are developed which modeled real-world problem in mathematics, biology, engineering, economics, physics, and other areas of science and technology [20–23]. In fractional calculus, a variety of fractional operators are introduced for the study of real-world issues. These operators, on the other hand, have a power law kernel and can only simulate physical problems to a limited extent. To solve these challenges and limitations, Caputo and Fabrizio presented a new fractional operator with an exponential decay kernel. Because of its nonsingular kernel, this unique operator is a revolutionary fractional derivative operator that has piqued the interest of many scholars. The results of this novel operator are more suitable and have many applications [24, 25]. To be more specific, the transmission phenomena of cancer with treatment and unknown parameters have been successfully represented through CF derivative [26, 27]. To get more realistic findings, we choose to depict the transmission mechanism of breast cancer with side effects on patient heart during chemotherapy through CF fractional derivative.

These accurate results and outcomes of fractional calculus motivate us to inspect and interrogate the dynamics of breast cancer with adverse reactions of chemotherapy treatment on patient heart through Caputo-Fabrizio (CF) fractional operator. In Section 1 of the article, we represent the fundamental idea of fractional calculus for the analysis of our system. In Section 2, a fractional model is formulated for breast cancer with the adverse reactions of chemotherapy treatment on the heart of a patient in fractional framework. The proposed model of breast cancer is then investigated through mathematical skills. The existence and uniqueness of the solution of the formulated FO model of breast cancer patients through the fixed point theorem are presented in Section 3 of the article. The dynamics of proposed cancer model is then analyzed with the variation of different input parameters numerically in Section 4. Finally, concluding remarks and suggestions are presented in the last section.

## 2. Formulation of the Model

In the formulation of the model, we consider the population of breast cancer patients in a hospital where we categorized the total population of breast cancer patient into stage 1, stage 2, stage 3, and stage 4 subpopulations during the first medical report. It is assumed that all the patient are treated with chemotherapy treatment in the hospital where the patients are passing with different stages during treatment, some patients experience cardiotoxicity, and some patients experience recovery while some getting worse condition of the disease during chemotherapy process. A compartmental model of five subgroups is formulated having subcompartments of stages 1 and 2 (*𝒞*_*A*_), stage 3 (*𝒞*_*B*_), stage 4 (*𝒞*_*C*_), disease-free state (*𝒞*_*D*_), and cardiotoxic (*𝒞*_*E*_) subgroups where the number of cancer patients in stages 1 and 2 is smaller than the other stages; therefore, they are placed in one subgroup.

New patients identified to suffer in stages 1 and 2 cancer are assumed to be *η*_1_ while for stage 3 and stage 4 are assumed to be *η*_2_ and *η*_3_, respectively. The subgroup *𝒞*_*A*_ having chemotherapy may either move worse subgroup *𝒞*_*B*_ with *δ*_*AB*_ or recover with a rate *δ*_*AD*_. The patients of the subgroup *𝒞*_*B*_ who are first treated in the hospital are recruited with a rate *η*_2_. This subgroup is more intensive chemotherapy as compares to *𝒞*_*A*_, where the patient die from cancer with a rate *γ*_2_, move to the recover subgroup with a rate *δ*_*BD*_, become more worse with a rate *δ*_*BC*_, and at a rate *δ*_*BE*_ become cardiotoxicity. The patients of cancer are recruited to subgroup *𝒞*_*C*_ with a rate *η*_3_ during the treatment. In this case, the rate of recovery *δ*_*CD*_ is smaller than the first two and rate *δ*_*CE*_ towards cardiotoxicity is greater than the rate of the subgroup *𝒞*_*B*_ due to intensive chemotherapy effect. We assume *γ*_3_ to be the death rate of cancer patient in this subgroup. In the forth subgroup, the population increased from the first three subgroups and lose recovery at *δ*_*DB*_, *δ*_*DC*_, and *δ*_*DE*_ to the subgroups *𝒞*_*B*_, *𝒞*_*C*_, and *𝒞*_*E*_, respectively. The patient in (*𝒞*_*E*_) comes from (*𝒞*_*B*_), (*𝒞*_*C*_) and (*𝒞*_*D*_) and taste cardiac death with rate*γ*_1_. Then, the dynamics of breast cancer with chemotherapy treatment with the above assumptions is given by the following system of ODEs:

(1) $$\begin{array}{c} \left\{\begin{array}{c} \frac{dC_{A}}{dt}=\eta_{1}-\delta_{AD}C_{A}-\delta_{AB}C_{A},\\ \frac{dC_{B}}{dt}=\eta_{2}+\delta_{AB}C_{A}+\delta_{DB}C_{D}-\delta_{BD}C_{B}-\delta_{BC}C_{B}-\delta_{BE}C_{B}-\gamma_{2}C_{B},\\ \frac{dC_{C}}{dt}=\eta_{3}+\delta_{BC}C_{B}+\delta_{DC}C_{D}-\delta_{CD}C_{C}-\delta_{CE}C_{C}-\gamma_{3}C_{C},\\ \frac{dC_{D}}{dt}=\delta_{AD}C_{A}+\delta_{BD}C_{B}+\delta_{CD}C_{C}-\delta_{DB}C_{D}-\delta_{DC}C_{D}-\delta_{DE}C_{D},\\ \frac{dC_{E}}{dt}=\delta_{DE}C_{D}+\delta_{CE}C_{C}+\delta_{BE}C_{B}-\gamma_{1}C_{E}, \end{array}\right. \end{array}$$

with appropriate initial condition for vector

(2) $$\begin{array}{c} C_{A}\left(0\right)\geq 0,C_{B}\left(0\right)\geq 0,C_{C}\left(0\right)\geq 0,C_{D}\left(0\right)\geq 0,C_{E}\left(0\right)\geq 0. \end{array}$$

It is well-know that fractional system provides more accurate results of the dynamics of a system developed from natural phenomena. There are several fractional operators in the literature of fractional calculus with power law kernel and have limitations to mimic real-world problems. Therefore, we applied Caputo-Fabrizio operator to our problem which represents the dynamics of mathematical model through exponential decay kernel to overcome these challenges and limitations. The dynamics of breast cancer through CF fractional derivative can be expressed as follows:

(3) D0CFtϑht=Uϑ1−ϑ∫ath′xexp−ϑt−x1−ϑdx.

A detailed discussion of this operator has been presented in the upcoming section of the article. We represent the system (1) of breast cancer with the help of the above definition of CF derivative as

(4) D0CFtϑCA=η1−δADCA−δABCA,D0CFtϑCB=η2+δABCA+δDBCD−δBDCB−δBCCB−δBECB−γ2CB,D0CFtϑCC=η3+δBCCB+δDCCD−δCDCC−δCECC−γ3CC,D0CFtϑCD=δADCA+δBDCB+δCDCC−δDBCD−δDCCD−δDECD,D0CFtϑCE=δDECD+δCECC+δBECB−γ1CE,

where *ϑ* is the order of CF fractional derivative such that 0 < *ϑ* ≤ 1 and the unit of the above fractional system is [*ϑ*]^−1^. In the next subsection, we will list some basic definitions and statements related to CF fractional derivative for further analysis of the model.

### 2.1. Rudimentary Knowledge

In this subsection of the article, the fundamental results and definitions of fractional Caputo-Fabrizio (CF) is presented for the analysis of our breast cancer model with chemotherapy treatment. The basic definitions and results are given below:

**Definition 1 .**

Let us suppose *h* ∈ *H*^1^(*a*, *b*), where *b* is greater than *a*; then, the CF derivative [28] of order *ϑ* is given by

(5) $$\begin{array}{c} D_{t}^{\vartheta }\left(h\left(t\right)\right)=\frac{U\left(\vartheta \right)}{1-\vartheta }\int_{a}^{t}h^{\prime }\left(x\right)\exp\left[-\vartheta \frac{t-x}{1-\vartheta }\right]dx, \end{array}$$

where *ϑ* ∈ [0, 1] and *U*(*τ*) denotes normality with *U*(0) = *U*(1) = 1 [28]. In the case, when *h* ∉ *H*^1^(*a*, *b*), then the following fractional derivative is obtained:

(6) $$\begin{array}{c} D_{t}^{\vartheta }\left(h\left(t\right)\right)=\frac{\vartheta U\left(\vartheta \right)}{1-\vartheta }\int_{a}^{t}\left(h\left(t\right)-h\left(x\right)\right)\exp\;\left[-\vartheta \frac{t-x}{1-\vartheta }\right]dx. \end{array}$$

**Remark 1 .**

Let us take *α* = 1 − *ϑ*/*ϑ* ∈ [0, ∞) and *ϑ* = 1/1 + *α* ∈ [0, 1]; then, equation (6) can be written in the following form:

(7) $$\begin{array}{c} D_{t}^{\vartheta }\left(h\left(t\right)\right)=\frac{M\left(\alpha \right)}{\alpha }\int_{a}^{t}h^{\prime }\left(x\right)e^{\left[-\frac{t-x}{\alpha }\right]}dx,M\left(0\right)=M\left(\infty \right)=1. \end{array}$$

Furthermore,

(8) $$\begin{array}{c} \underset{\alpha ⟶0}{\lim}\frac{1}{\alpha }\exp\left[-\frac{t-x}{\alpha }\right]=\delta \left(x-t\right). \end{array}$$

In [29], the authors introduced the concept of fractional integral which is defined as follows:

**Definition 2 .**

Let *h* be a given function; then, the fractional integral is defined in the following manner:

(9) $$\begin{array}{c} I_{t}^{\vartheta }\left(h\left(t\right)\right)=\frac{2\left(1-\vartheta \right)}{\left(2-\vartheta \right)U\left(\vartheta \right)}h\left(t\right)+\frac{2\vartheta }{\left(2-\vartheta \right)U\left(\vartheta \right)}\int_{0}^{t}h\left(u\right)du,t\geq 0, \end{array}$$

where 0 < *ϑ* < 1 is the order of the above fractional integral.

**Remark 2 .**

From the above Definition 3, we can conclude that

(10) $$\begin{array}{c} \frac{2\left(1-\vartheta \right)}{\left(2-\vartheta \right)U\left(\vartheta \right)}+\frac{2\vartheta }{\left(2-\vartheta \right)U\left(\vartheta \right)}=1, \end{array}$$

which gives *U*(*ϑ*) = 2/2 − *ϑ*, 0 < *ϑ* < 1. A new Caputo derivative of order *ϑ* was introduced by Losada and Nieto in [29] by using equation (10) and is given by

(11) $$\begin{array}{c} D_{t}^{\vartheta }\left(h\left(t\right)\right)=\frac{1}{1-\vartheta }\int_{0}^{t}h^{\prime }\left(x\right)\exp\left[\vartheta \frac{t-x}{1-\vartheta }\right]dx,0<\vartheta <1. \end{array}$$

For the equilibrium point of breast cancer model (4), we set all the fractional derivative of model (4) to zero and obtain the equilibrium point given by *ℰ*_*e*_ = (*𝒞*_*A*_^∗^, *𝒞*_*B*_^∗^, *𝒞*_*C*_^∗^, *𝒞*_*D*_^∗^, *𝒞*_*E*_^∗^). The equilibrium point exists and is

(12) $$\begin{array}{c} C_{A}^{*}=\frac{\eta_{1}}{k_{1}},C_{B}^{*}=\frac{\alpha }{k_{1}\lambda },C_{C}^{*}=\frac{\beta }{k_{1}\lambda },\\ C_{D}^{*}=\frac{\xi }{k_{1}\lambda },\\ C_{E}^{*}=\frac{v}{k_{1}\lambda \gamma_{1}}, \end{array}$$

where,

(13) $$\begin{array}{c} \alpha =\left(k_{3}\delta_{BD}+\left(\delta_{DE}+\delta_{DC}\right)\gamma_{3}+\left(\delta_{DE}+\delta_{DC}\right)\delta_{CE}+\delta_{DE}\delta_{CD}\right)\eta_{2}\delta_{AB}+\left(k_{3}\eta_{1}+\delta_{CD}\eta_{3}\right)\delta_{DB}+\eta_{1}\left(\delta_{DE}+\delta_{DC}\right)\gamma_{3}+\left(\delta_{DE}+\delta_{DC}\right)\delta_{CE}+\left.\delta_{DE}\delta_{CD}\right)\delta_{AB}+\delta_{AD}\left(\left(k_{3}\delta_{DB}+\left(\delta_{DE}+\delta_{DC}\right)\gamma_{3}+\left(\delta_{DE}+\delta_{DC}\right)\delta_{CE}+\delta_{DE}\delta_{CD}\right)\eta_{2}+\left(k_{3}\eta_{1}+\delta_{CD}\eta_{3}\right)\delta_{DB}\right),\\ \beta =\left(k_{2}\delta_{DC}+\left(\delta_{DB}+\delta_{DE}\right)\delta_{BC}+\left(\gamma_{2}+\delta_{BD}+\delta_{BE}\right)\delta_{DE}+\delta_{DB}\left(\gamma_{2}+\delta_{BE}\right)\right)k_{1}\eta_{3}+\left(\left(\left(\eta_{1}+\eta_{2}\right)\delta_{BC}+\left(\gamma_{2}+\delta_{BD}+\delta_{BE}\right)\eta_{1}+\delta_{BD}\eta_{2}\right)\delta_{DC}+\left(\eta_{2}\delta_{DE}+\delta_{DB}\left(\eta_{1}+\eta_{2}\right)\right)\delta_{BC}\right)\delta_{AD}+\left(\left(\delta_{BC}+\delta_{BD}\right)\delta_{DC}+\left(\delta_{DB}+\delta_{DE}\right)\delta_{BC}\right)\left(\eta_{1}+\eta_{2}\right)\delta_{AB},\\ \xi =\left(\left(k_{2}\eta_{1}+\left(\eta_{1}+\eta_{3}\right)\right.\delta_{BD}+\delta_{BC}\eta_{2}+\eta_{3}\left(\gamma_{2}+\delta_{BC}+\delta_{BE}\right)\delta_{CD}+\left(\left(k_{2}\eta_{1}+\delta_{BD}\eta_{2}\right)\left(\gamma_{3}+\delta_{CE}\right)\right)\right)\delta_{AD}+\delta_{AB}\left(\left(\delta_{BC}+\delta_{BD}\right)\eta_{1}+\left(\eta_{2}+\eta_{3}\right)\delta_{BD}+\delta_{BC}\eta_{2}+\eta_{3}\left(\gamma_{2}+\delta_{BC}+\delta_{BE}\right)\delta_{CD}+\delta_{BD}\left(\eta_{1}+\eta_{2}\right)\left(\gamma_{3}+\delta_{CE}\right)\right),\\ v=\left(\left(\eta_{1}+\eta_{2}+\eta_{3}\right)\delta_{BE}+\left(\gamma_{2}+\delta_{BC}+\delta_{BD}\right)\eta_{1}+\left(\delta_{BC}+\delta_{BD}\right)\eta_{2}+\eta_{3}\left(\gamma_{2}+\delta_{BC}+\delta_{BD}\right)\right)\delta_{DE}\delta_{AD}\delta_{CE}+\left(\delta_{DB}+\delta_{DC}\right)\left(\eta_{1}+\eta_{2}+\eta_{3}\right)\delta_{BE}+\left(\left(\delta_{DB}+\delta_{DC}\right)\delta_{BC}+\delta_{DC}\left(\gamma_{2}+\delta_{BD}\right)\eta_{1}+\left(\left(\delta_{BD}+\delta_{DC}\right)\delta_{BC}+\delta_{BD}\delta_{DC}\right)\eta_{2}+\left(\left(\delta_{DB}+\delta_{DC}\right)\delta_{BC}+\gamma_{2}\delta_{DB}+\delta_{DC}\left(\gamma_{2}+\delta_{BD}\right)\right)\eta_{3}\delta_{AD}\delta_{CE}+\left(\left(\left(\eta_{+}\eta_{2}+\eta_{3}\right)\delta_{BE}+\left(\delta_{BC}+\delta_{BD}\right)\eta_{1}+\left(\delta_{BC}+\delta_{BD}\right)\eta_{2}+\eta_{3}\left(\gamma_{2}+\delta_{BC}+\delta_{BD}\right)\right)\delta_{DE}\right)\delta_{AB}\delta_{CE}+\left(\left(\delta_{DB}+\delta_{DC}\right)\left(\eta_{1}+\eta_{2}+\eta_{3}\right)\delta_{BE}+\left(\delta_{DB}+\delta_{DC}\right)\delta_{BC}+\delta_{BD}\delta_{DC}\right)\eta_{1}\right)\delta_{AB}\delta_{CE}+\left(\left(\left(\delta_{DB}+\delta_{DC}\right)\delta_{BC}+\delta_{BD}\delta_{DC}\right)\eta_{2}+\left(\left(\delta_{DB}+\delta_{DC}\right)\delta_{BC}+\gamma_{2}\delta_{DB}+\delta_{DC}\left(\gamma_{2}+\delta_{BD}\right)\right)\eta_{3}\right)\delta_{AB}\delta_{CE}+\delta_{DE}\delta_{AD}\left(\left(\left(\gamma_{3}+\delta_{CD}\right)\eta_{1}+\left(\gamma_{3}+\delta_{CD}\right)\eta_{2}+\eta_{3}\delta_{CD}\right)\delta_{BE}+\left(\gamma_{3}+\delta_{CD}\right)\left(\gamma_{2}+\delta_{BC}+\delta_{BD}\right)\right)\eta_{1}+\left(\left(\left(\delta_{BC}+\delta_{BD}\right)\delta_{DC}+\gamma_{3}\delta_{BD}\right)\eta_{2}+\eta_{3}\delta_{CD}\left(\gamma_{2}+\delta_{BC}+\delta_{BD}\right)\right)\delta_{DE}\delta_{AD}+\delta_{BE}\left(\left(\gamma_{3}+\delta_{CD}\right)\delta_{DB}\eta_{1}+\left(\delta_{DB}\delta_{CD}+\gamma_{3}\left(\delta_{DB}+\delta_{DC}\right)\right)\eta_{2}+\eta_{3}\delta_{CD}\delta_{DB}\right)\delta_{AD}+\delta_{AB}\delta_{DE}\left(\left(\left(\gamma_{3}+\delta_{CD}\right)\eta_{1}+\left(\gamma_{3}+\delta_{CD}\right)\eta_{2}+\eta_{3}\delta_{CD}\right)\delta_{BE}\left(\left(\delta_{BC}+\delta_{BD}\right)\delta_{CD}+\gamma_{3}\delta_{BD}\right)\eta_{1}\right)+\delta_{AB}\delta_{DE}\left(\left(\left(\delta_{BC}+\delta_{BD}\right)\delta_{CD}+\gamma_{3}\delta_{BD}\right)\eta_{2}+\eta_{3}\delta_{CD}\left(\gamma_{2}+\delta_{BC}+\delta_{BD}\right)\right)+\delta_{BE}\delta_{AB}\left(\left(\delta_{BD}\delta_{CD}+\gamma_{3}\left(\delta_{DB}+\delta_{DC}\right)\eta_{1}+\left(\left(\delta_{DB}\delta_{CD}+\gamma_{3}\left(\delta_{BD}+\delta_{DC}\right)\right.\right.\right)\eta_{2}+\eta_{3}\delta_{CD}\delta_{DB}\right),\\ \lambda =k_{1}k_{2}\delta_{DE}+\left(\left(\delta_{DB}+\delta_{DC}\right)\gamma_{2}+\left(\delta_{DB}+\delta_{DC}\right)\delta_{BE}+\delta_{BC}\delta_{DB}+\left(\delta_{BC}+\delta_{BD}\right)\delta_{DC}\right)\gamma_{3}+\left(\left(\delta_{DB}+\delta_{DC}\right)\gamma_{2}+\left(\delta_{DB}+\delta_{DC}\right)\delta_{BE}+\delta_{BC}\delta_{DB}+\left(\delta_{BC}+\delta_{BD}\right)\delta_{DC}\right)\delta_{CE}+\delta_{CD}\delta_{DB}\left(\gamma_{2}+\delta_{BE}\right), \end{array}$$

in which *k*_1_ = *δ*_*AD*_ + *δ*_*AB*_, *k*_2_ = *δ*_*BD*_ + *δ*_*BC*_ + *δ*_*BE*_ + *γ*_2_, and *k*_3_ = *δ*_*CD*_ + *δ*_*CE*_ + *γ*_3_. Here, for equilibrium of our fractional-order breast cancer model, we have the following conclusion. The disease-free equilibrium point can be easily determined by taking the steady state of our system without infection. These equilibrium points are important for the analysis of the proposed fractional model of cancer with chemotherapy treatment and can predict sufficient condition for the control and spread of the infection. We have the following result based on the above investigation:

**Theorem 1 .**

There exists an equilibrium of the proposed fractional model (4) of breast cancer without any condition.

## 3. Interrogation of Fractional System

Here, the solution of the proposed breast cancer model will be investigated for existence through fixed point theory. We use the concept of CF fractional derivative on the system (4) and get the following:

(14) CAt−CA0=I0CFtϑη1−δADCA−δABCA,CBt−CB0=I0CFtϑη2+δABCA+δDBCD−δBDCB−δBCCB−δBECB−γ2CB,CCt−CC0=I0CFtϑη3+δBCCB+δDCCD−δCDCC−δCECC−γ3CC,cCDt−CD0=I0CFtϑδADCA+δBDCB+δCDCC−δDBCD−δDCCD−δDECD,CEt−CE0=I0CFtϑδDECD+δCECC+δBECB−γ1CE.

By applying the idea presented in [29], we get

(15) $$\begin{array}{c} C_{A}\left(t\right)-C_{A}\left(0\right)=\frac{2\left(1-\vartheta \right)}{\left(2-\vartheta \right)U\left(\vartheta \right)}\left[\eta_{1}-\delta_{AD}C_{A}-\delta_{AB}C_{A}\right]+\frac{2\vartheta }{\left(2-\vartheta \right)U\left(\vartheta \right)}\int_{0}^{t}\left[\eta_{1}-\delta_{AD}C_{A}-\delta_{AB}C_{A}\right]dy, \end{array}$$

(16) $$\begin{array}{c} C_{B}\left(t\right)-C_{B}\left(0\right)=\frac{2\left(1-\vartheta \right)}{\left(2-\vartheta \right)U\left(\vartheta \right)}\left[\eta_{2}+\delta_{AB}C_{A}+\delta_{DB}C_{D}-\delta_{BD}C_{B}-\delta_{BC}C_{B}-\delta_{BE}C_{B}-\gamma_{2}C_{B}\right]+\frac{2\vartheta }{\left(2-\vartheta \right)U\left(\vartheta \right)}\int_{0}^{t}\left[\eta_{2}+\delta_{AB}C_{A}+\delta_{DB}C_{D}-\delta_{BD}C_{B}-\delta_{BC}C_{B}-\delta_{BE}C_{B}-\gamma_{2}C_{B}\right]dy, \end{array}$$

(17) $$\begin{array}{c} C_{C}\left(t\right)-C_{C}\left(0\right)=\frac{2\left(1-\vartheta \right)}{\left(2-\vartheta \right)U\left(\vartheta \right)}\left[\eta_{3}+\delta_{BC}C_{B}+\delta_{DC}C_{D}-\delta_{CD}C_{C}-\delta_{CE}C_{C}-\gamma_{3}C_{C}\right]+\frac{2\vartheta }{\left(2-\vartheta \right)U\left(\vartheta \right)}\int_{0}^{t}\left[\eta_{3}+\delta_{BC}C_{B}+\delta_{DC}C_{D}-\delta_{CD}C_{C}-\delta_{CE}C_{C}-\gamma_{3}C_{C}\right]dy, \end{array}$$

(18) $$\begin{array}{c} C_{D}\left(t\right)-C_{D}\left(0\right)=\frac{2\left(1-\vartheta \right)}{\left(2-\vartheta \right)U\left(\vartheta \right)}\left[\delta_{AD}C_{A}+\delta_{BD}C_{B}+\delta_{CD}C_{C}-\delta_{DB}C_{D}-\delta_{DC}C_{D}-\delta_{DE}C_{D}\right]+\frac{2\vartheta }{\left(2-\vartheta \right)U\left(\vartheta \right)}\int_{0}^{t}\left[\delta_{AD}C_{A}+\delta_{BD}C_{B}+\delta_{CD}C_{C}-\delta_{DB}C_{D}-\delta_{DC}C_{D}-\delta_{DE}C_{D}\right]dy, \end{array}$$

(19) $$\begin{array}{c} C_{E}\left(t\right)-C_{E}\left(0\right)=\frac{2\left(1-\vartheta \right)}{\left(2-\vartheta \right)U\left(\vartheta \right)}\left[\delta_{DE}C_{D}+\delta_{CE}C_{C}+\delta_{BE}C_{B}-\gamma_{1}C_{E}\right]+\frac{2\vartheta }{\left(2-\vartheta \right)U\left(\vartheta \right)}\int_{0}^{t}\left[\delta_{DE}C_{D}+\delta_{CE}C_{C}+\delta_{BE}C_{B}-\gamma_{1}C_{E}\right]. \end{array}$$

In the next step, we proceed in the following manner:

(20) $$\begin{array}{c} \left\{\begin{array}{c} L_{1}\left(t,C_{A}\right)=\eta_{1}-\delta_{AD}C_{A}-\delta_{AB}C_{A},\\ L_{2}\left(t,C_{B}\right)=\eta_{2}+\delta_{AB}C_{A}+\delta_{DB}C_{D}-\delta_{BD}C_{B}-\delta_{BC}C_{B}-\delta_{BE}C_{B}-\gamma_{2}C_{B},\\ L_{3}\left(t,C_{C}\right)=\eta_{3}+\delta_{BC}C_{B}+\delta_{DC}C_{D}-\delta_{CD}C_{C}-\delta_{CE}C_{C}-\gamma_{3}C_{C},\\ L_{4}\left(t,C_{D}\right)=\delta_{AD}C_{A}+\delta_{BD}C_{B}+\delta_{CD}C_{C}-\delta_{DB}C_{D}-\delta_{DC}C_{D}-\delta_{DE}C_{D},\\ L_{5}\left(t,C_{E}\right)=\delta_{DE}C_{D}+\delta_{CE}C_{C}+\delta_{BE}C_{B}-\gamma_{1}C_{E}. \end{array}\right. \end{array}$$

**Theorem 2 .**

If the following condition satisfies

(21) $$\begin{array}{c} 0\leq \left(\delta_{AD}+\delta_{AB}\right)<1, \end{array}$$

then, the kernels *ℒ*_1_, *ℒ*_2_, *ℒ*_3_, *ℒ*_4_, and *ℒ*_5_ assure the Lipschitz condition.

**Proof**

For the proof of Theorem 7, we first take *𝒞*_*A*_ and *𝒞*_*A*1_ and start from *ℒ*_1_ in the following manner:

(22) $$\begin{array}{c} L_{1}\left(t,C_{A}\right)-L_{1}\left(t,C_{A1}\right)=-\delta_{AD}C_{A}+\delta_{AD}C_{A1}-\delta_{AB}C_{A}+\delta_{AB}C_{A1}. \end{array}$$

Here, apply norm on Eq. (19) and simplify; we get the following:

(23) $$\begin{array}{c} \left\|L_{1}\left(t,C_{A}\right)-L_{1}\left(t,C_{A1}\right)\right\|\leq \left\|-\delta_{AD}C_{A}+\delta_{AD}C_{A1}\right\|+\left\|-\delta_{AB}C_{A}+\delta_{AB}C_{A1}\right\|\leq \delta_{AD}\left\|C_{A}-C_{A1}\right\|+\delta_{AB}\left\|C_{A}-C_{A1}\right\|\leq \left(\delta_{AD}+\delta_{AB}\right)\left\|C_{A}-C_{A1}\right\|. \end{array}$$

At this stage, we assume *μ*_1_ = (*δ*_*AD*_ + *δ*_*AB*_); then, the following result is obtained:

(24) $$\begin{array}{c} \left\|L_{1}\left(t,C_{A}\right)-L_{1}\left(t,{C_{A}}_{1}\right)\right\|\leq \mu_{1}\left\|C_{A}\left(t\right)-C_{A}\left(t_{1}\right)\right\|. \end{array}$$

Thus, the Lipschitz condition is fulfilled for *ℒ*_1_; in addition to this, the condition 0 ≤ (*δ*_*AD*_ + *δ*_*AB*_) < 1 assure that the contraction is also satisfied. In the same way, the Lipschitz conditions for the other cases of our system are determined as

(25) $$\begin{array}{c} \left\|L_{2}\left(t,C_{B}\right)-L_{2}\left(t,C_{B1}\right)\right\|\leq \mu_{2}\left\|C_{B}\left(t\right)-C_{B}\left(t_{1}\right)\right\|,\\ \left\|L_{3}\left(t,C_{C}\right)-L_{3}\left(t,C_{C1}\right)\right\|\leq \mu_{3}\left\|C_{C}\left(t\right)-C_{C}\left(t_{1}\right)\right\|,\\ \left\|L_{4}\left(t,C_{D}\right)-L_{4}\left(t,C_{D1}\right)\right\|\leq \mu_{4}\left\|C_{D}\left(t\right)-C_{D}\left(t_{1}\right)\right\|,\\ \left\|L_{5}\left(t,C_{E}\right)-L_{5}\left(t,C_{E1}\right)\right\|\leq \mu_{5}\left\|C_{E}\left(t\right)-C_{E}\left(t_{1}\right)\right\|. \end{array}$$

Further simplification of Eq. (19) implies

(26) $$\begin{array}{c} \left\{\begin{array}{c} C_{A}\left(t\right)=C_{A}\left(t\right)\left(0\right)+\frac{2\left(1-\vartheta \right)}{\left(2-\vartheta \right)U\left(\vartheta \right)}L_{1}\left(t,C_{A}\left(t\right)\right)+\frac{2\vartheta }{\left(2-\vartheta \right)U\left(\vartheta \right)}\int_{0}^{t}\left(L_{1}\left(y,C_{A}\left(t\right)\right)\right)dy,\\ C_{B}\left(t\right)=C_{B}\left(t\right)\left(0\right)+\frac{2\left(1-\vartheta \right)}{\left(2-\vartheta \right)U\left(\vartheta \right)}L_{2}\left(t,C_{B}\left(t\right)\right)+\frac{2\vartheta }{\left(2-\vartheta \right)U\left(\vartheta \right)}\int_{0}^{t}\left(L_{2}\left(y,C_{B}\left(t\right)\right)\right)dy,\\ C_{C}\left(t\right)=C_{C}\left(t\right)\left(0\right)+\frac{2\left(1-\vartheta \right)}{\left(2-\vartheta \right)U\left(\vartheta \right)}L_{3}\left(t,C_{B}\left(t\right)\right)+\frac{2\vartheta }{\left(2-\vartheta \right)U\left(\vartheta \right)}\int_{0}^{t}\left(L_{3}\left(y,C_{C}\left(t\right)\right)\right)dy,\\ C_{D}\left(t\right)=C_{D}\left(t\right)\left(0\right)+\frac{2\left(1-\vartheta \right)}{\left(2-\vartheta \right)U\left(\vartheta \right)}L_{4}\left(t,C_{D}\left(t\right)\right)+\frac{2\vartheta }{\left(2-\vartheta \right)U\left(\vartheta \right)}\int_{0}^{t}\left(L_{4}\left(y,C_{D}\left(t\right)\right)\right)dy,\\ C_{E}\left(t\right)=C_{E}\left(t\right)\left(0\right)+\frac{2\left(1-\vartheta \right)}{\left(2-\vartheta \right)U\left(\vartheta \right)}L_{5}\left(t,C_{E}\left(t\right)\right)+\frac{2\vartheta }{\left(2-\vartheta \right)U\left(\vartheta \right)}\int_{0}^{t}\left(L_{5}\left(y,C_{E}\left(t\right)\right)\right)dy. \end{array}\right. \end{array}$$

Its recursive form is given by

(27) $$\begin{array}{c} \left\{\begin{array}{c} C_{\text{An}}\left(t\right)=2\frac{\left(1-\vartheta \right)}{\left(2-\vartheta \right)U\left(\vartheta \right)}L_{1}\left(t,C_{A\left(n-1\right)}\right)+2\frac{\vartheta }{\left(2-\vartheta \right)U\left(\vartheta \right)}\int_{0}^{t}\left(L_{1}\left(y,C_{A\left(n-1\right)}\right)\right)dy,\\ C_{Bn}\left(t\right)=2\frac{\left(1-\vartheta \right)}{\left(2-\vartheta \right)U\left(\vartheta \right)}L_{2}\left(t,C_{B\left(n-1\right)}\right)+2\frac{\vartheta }{\left(2-\vartheta \right)U\left(\vartheta \right)}\int_{0}^{t}\left(L_{2}\left(y,C_{B\left(n-1\right)}\right)\right)dy,\\ C_{Cn}\left(t\right)=2\frac{\left(1-\vartheta \right)}{\left(2-\vartheta \right)U\left(\vartheta \right)}L_{3}\left(t,C_{C\left(n-1\right)}\right)+2\frac{\vartheta }{\left(2-\vartheta \right)U\left(\vartheta \right)}\int_{0}^{t}\left(L_{3}\left(y,C_{C\left(n-1\right)}\right)\right)dy,\\ C_{Dn}\left(t\right)=2\frac{\left(1-\vartheta \right)}{\left(2-\vartheta \right)U\left(\vartheta \right)}L_{4}\left(t,C_{D\left(n-1\right)}\right)+2\frac{\vartheta }{\left(2-\vartheta \right)U\left(\vartheta \right)}\int_{0}^{t}\left(L_{4}\left(y,C_{D\left(n-1\right)}\right)\right)dy,\\ C_{En}\left(t\right)=2\frac{\left(1-\vartheta \right)}{\left(2-\vartheta \right)U\left(\vartheta \right)}L_{5}\left(t,C_{E\left(n-1\right)}\right)+2\frac{\vartheta }{\left(2-\vartheta \right)U\left(\vartheta \right)}\int_{0}^{t}\left(L_{5}\left(y,C_{E\left(n-1\right)}\right)\right)dy, \end{array}\right. \end{array}$$

with proper initial conditions

(28) $$\begin{array}{c} C_{A}^{0}\left(t\right)=C_{A}\left(0\right),C_{B}^{0}\left(t\right)=C_{B}\left(0\right),C_{C}^{0}\left(t\right)=C_{C}\left(0\right),C_{D}^{0}\left(t\right)=C_{D}\left(0\right),C_{E}^{0}\left(t\right)=C_{E}\left(0\right). \end{array}$$

Here, the succeeding difference form is

(29) $$\begin{array}{c} \hbar_{1n}\left(t\right)=C_{\text{An}}\left(t\right)-{C_{A}}_{\left(n-1\right)}\left(t\right)=\frac{2\left(1-\vartheta \right)}{\left(2-\vartheta \right)U\left(\vartheta \right)}\left(L_{1}\left(t,C_{A\left(n-1\right)}\right)-L_{1}\left(t,C_{A\left(n-2\right)}\right)\right)+2\frac{\vartheta }{\left(2-\vartheta \right)U\left(\vartheta \right)}\int_{0}^{t}\left(L_{1}\left(y,{C_{A}}_{\left(n-1\right)}\right)-L_{1}\left(y,{C_{A}}_{\left(n-2\right)}\right)\right)dy,\\ \hbar_{2n}\left(t\right)=C_{Bn}\left(t\right)-{C_{B}}_{\left(n-1\right)}\left(t\right)=\frac{2\left(1-\vartheta \right)}{\left(2-\vartheta \right)U\left(\vartheta \right)}\left(L_{2}\left(t,C_{B\left(n-1\right)}\right)-L_{2}\left(t,C_{B\left(n-2\right)}\right)\right)+2\frac{\vartheta }{\left(2-\vartheta \right)U\left(\vartheta \right)}\int_{0}^{t}\left(L_{2}\left(y,{C_{B}}_{\left(n-1\right)}\right)-L_{2}\left(y,{C_{B}}_{\left(n-2\right)}\right)\right)dy,\\ \hbar_{3n}\left(t\right)=C_{Cn}\left(t\right)-{C_{C}}_{\left(n-1\right)}\left(t\right)=\frac{2\left(1-\vartheta \right)}{\left(2-\vartheta \right)U\left(\vartheta \right)}\left(L_{3}\left(t,C_{C\left(n-1\right)}\right)-L_{3}\left(t,C_{C\left(n-2\right)}\right)\right)+2\frac{\vartheta }{\left(2-\vartheta \right)U\left(\vartheta \right)}\int_{0}^{t}\left(L_{3}\left(y,{C_{C}}_{\left(n-1\right)}\right)-L_{3}\left(y,{C_{C}}_{\left(n-2\right)}\right)\right)dy,\\ \hbar_{4n}\left(t\right)=C_{Dn}\left(t\right)-{C_{D}}_{\left(n-1\right)}\left(t\right)=\frac{2\left(1-\vartheta \right)}{\left(2-\vartheta \right)U\left(\vartheta \right)}\left(L_{4}\left(t,C_{D\left(n-1\right)}\right)-L_{4}\left(t,C_{D\left(n-2\right)}\right)\right)+2\frac{\vartheta }{\left(2-\vartheta \right)U\left(\vartheta \right)}\int_{0}^{t}\left(L_{4}\left(y,{C_{D}}_{\left(n-1\right)}\right)-L_{4}\left(y,{C_{D}}_{\left(n-2\right)}\right)\right)dy,\\ \hbar_{5n}\left(t\right)=C_{En}\left(t\right)-{C_{E}}_{\left(n-1\right)}\left(t\right)=\frac{2\left(1-\vartheta \right)}{\left(2-\vartheta \right)U\left(\vartheta \right)}\left(L_{5}\left(t,C_{E\left(n-1\right)}\right)-L_{5}\left(t,C_{E\left(n-2\right)}\right)\right)+2\frac{\vartheta }{\left(2-\vartheta \right)U\left(\vartheta \right)}\int_{0}^{t}\left(L_{5}\left(y,{C_{E}}_{\left(n-1\right)}\right)-L_{5}\left(y,{C_{E}}_{\left(n-2\right)}\right)\right)dy. \end{array}$$

Here, we observe the following:

(30) $$\begin{array}{c} \left\{\begin{array}{c} C_{\text{An}}\left(t\right)=\overset{n}{\underset{i=1}{\sum }}\hbar_{1i}\left(t\right),C_{Bn}\left(t\right)=\overset{n}{\underset{i=1}{\sum }}\hbar_{2i}\left(t\right),C_{Cn}\left(t\right)=\overset{n}{\underset{i=1}{\sum }}\hbar_{3i}\left(t\right),\\ C_{Dn}\left(t\right)=\overset{n}{\underset{i=1}{\sum }}\hbar_{4i}\left(t\right),C_{En}\left(t\right)=\overset{n}{\underset{i=1}{\sum }}\hbar_{5i}\left(t\right). \end{array}\right. \end{array}$$

Following the same way, we have

(31) $$\begin{array}{c} \left\|\hbar_{1n}\left(t\right)\right\|=\left\|C_{\text{An}}\left(t\right)-C_{A\left(n-1\right)}\left(t\right)\right\|=\left\|\begin{array}{c} \frac{\left(1-\vartheta \right)}{\left(2-\vartheta \right)U\left(\vartheta \right)}\left(L_{1}\left(t,C_{A\left(n-1\right)}\right)-L_{1}\left(t,C_{A\left(n-2\right)}\right)\right)\\ +2\frac{\vartheta }{\left(2-\vartheta \right)U\left(\vartheta \right)}\int_{0}^{t}\left(L_{1}\left(y,C_{A\left(n-1\right)}\right)-L_{1}\left(y,C_{A\left(n-2\right)}\right)\right)dy \end{array}\right\| \end{array}$$

By triangular inequality, Eq. (31) becomes

(32) $$\begin{array}{c} \left\|C_{\text{An}}\left(t\right)-C_{A\left(n-1\right)}\left(t\right)\right\|\leq 2\frac{\left(1-\vartheta \right)}{\left(2-\vartheta \right)U\left(\vartheta \right)}\left\|L_{1}\left(t,C_{A\left(n-1\right)}\right)-L_{1}\left(t,C_{A\left(n-2\right)}\right)\right\|+2\frac{\vartheta }{\left(2-\vartheta \right)U\left(\vartheta \right)}\left\|\;\int_{0}^{t}\left(L_{1}\left(y,C_{A\left(n-1\right)}\right)-L_{1}\left(y,C_{A\left(n-2\right)}\right)\right)dy\right\|. \end{array}$$

Lipschitz condition leads us to

(33) $$\begin{array}{c} \left\|{C_{A}}_{n}\left(t\right)-{C_{A}}_{n-1}\left(t\right)\right\|\leq 2\frac{\left(1-\vartheta \right)}{\left(2-\vartheta \right)U\left(\vartheta \right)}\mu_{1}\left\|C_{A\left(n-1\right)}-C_{A\left(n-2\right)}\right\|+2\frac{\vartheta }{\left(2-\vartheta \right)U\left(\vartheta \right)}\mu_{1}\times \int_{0}^{t}\left\|C_{A\left(n-1\right)}-C_{A\left(n-2\right)}\right\|dy. \end{array}$$

Next, we have

(34) $$\begin{array}{c} \left\|\hbar_{1n}\left(t\right)\right\|\leq 2\frac{\left(1-\vartheta \right)}{\left(2-\vartheta \right)U\left(\vartheta \right)}\mu_{1}\left\|\hbar_{1\left(n-1\right)}\left(t\right)\right\|+2\frac{\vartheta }{\left(2-\vartheta \right)U\left(\vartheta \right)}\mu_{1}\int_{0}^{t}\left\|\hbar_{1\left(n-1\right)}\left(y\right)\right\|dy. \end{array}$$

Taking the same steps, we get

(35) $$\begin{array}{c} \left\|\hbar_{2n}\left(t\right)\right\|\leq 2\frac{\left(1-\vartheta \right)}{\left(2-\vartheta \right)U\left(\vartheta \right)}\mu_{2}\left\|\hbar_{2\left(n-1\right)}\left(t\right)\right\|+2\frac{\vartheta }{\left(2-\vartheta \right)U\left(\vartheta \right)}\mu_{2}\int_{0}^{t}\left\|\hbar_{2\left(n-1\right)}\left(y\right)\right\|dy, \end{array}$$

(36) $$\begin{array}{c} \left\|\hbar_{3n}\left(t\right)\right\|\leq 2\frac{\left(1-\vartheta \right)}{\left(2-\vartheta \right)U\left(\vartheta \right)}\mu_{3}\left\|\hbar_{3\left(n-1\right)}\left(t\right)\right\|+2\frac{\vartheta }{\left(2-\vartheta \right)U\left(\vartheta \right)}\mu_{1}\int_{0}^{t}\left\|\hbar_{3\left(n-1\right)}\left(y\right)\right\|dy, \end{array}$$

(37) $$\begin{array}{c} \left\|\hbar_{4n}\left(t\right)\right\|\leq \frac{2\left(1-\vartheta \right)}{\left(2-\vartheta \right)U\left(\vartheta \right)}\mu_{4}\left\|\hbar_{4\left(n-1\right)}\left(t\right)\right\|+2\frac{\vartheta }{\left(2-\vartheta \right)U\left(\vartheta \right)}\mu_{4}\int_{0}^{t}\left\|\hbar_{4\left(n-1\right)}\left(y\right)\right\|dy, \end{array}$$

(38) $$\begin{array}{c} \left\|\hbar_{5n}\left(t\right)\right\|\leq 2\frac{\left(1-\vartheta \right)}{\left(2-\vartheta \right)U\left(\vartheta \right)}\mu_{5}\left\|\hbar_{5\left(n-1\right)}\left(t\right)\right\|+2\frac{\vartheta }{\left(2-\vartheta \right)U\left(\vartheta \right)}\mu_{5}\int_{0}^{t}\left\|\hbar_{5\left(n-1\right)}\left(y\right)\right\|dy. \end{array}$$

**Theorem 3 .**

Exact coupled solutions of the proposed breast cancer model (4) exists if the below mentioned condition satisfies. That is, one can find *t*_0_ in a way that

(39) $$\begin{array}{c} 2\frac{\left(1-\vartheta \right)}{\left(2-\vartheta \right)U\left(\vartheta \right)}\mu_{1}+2\frac{\vartheta }{\left(2-\vartheta \right)U\left(\vartheta \right)}\mu_{1}t_{0}<1. \end{array}$$

**Proof**

As the state variables *𝒞*_*A*_(*t*), *𝒞*_*B*_(*t*), *𝒞*_*C*_(*t*), *𝒞*_*D*_(*t*), and *𝒞*_*D*_(*t*) are bounded. Moreover, we have shown that the Lipschitz condition is fulfilled by the kernels; Eqs. (34) and (38) give the following by applying the recursive technique:

(40) $$\begin{array}{c} \left\|\hbar_{1n}\left(t\right)\right\|\leq \left\|C_{\text{An}}\left(0\right)\right\|{\left[\left(2\frac{\left(1-\vartheta \right)}{\left(2-\vartheta \right)U\left(\vartheta \right)}\mu_{1}\right)+\left(2\frac{\vartheta }{\left(2-\vartheta \right)U\left(\vartheta \right)}\mu_{1}t\right)\right]}^{n},\\ \left\|\hbar_{2n}\left(t\right)\right\|\left\|C_{Bn}\left(0\right)\right\|{\left[\left(2\frac{\left(1-\vartheta \right)}{\left(2-\vartheta \right)U\left(\vartheta \right)}\mu_{2}\right)+\left(2\frac{\vartheta }{\left(2-\vartheta \right)U\left(\vartheta \right)}\mu_{2}t\right)\right]}^{n},\\ \left\|\hbar_{3n}\left(t\right)\right\|\leq \left\|C_{Cn}\left(0\right)\right\|{\left[\left(2\frac{\left(1-\vartheta \right)}{\left(2-\vartheta \right)U\left(\vartheta \right)}\mu_{3}\right)+\left(2\frac{\vartheta }{\left(2-\vartheta \right)U\left(\vartheta \right)}\mu_{3}t\right)\right]}^{n},\\ \left\|\hbar_{4n}\left(t\right)\right\|\leq \left\|C_{Dn}\left(0\right)\right\|{\left[\left(2\frac{\left(1-\vartheta \right)}{\left(2-\vartheta \right)U\left(\vartheta \right)}\mu_{4}\right)+\left(2\frac{\vartheta }{\left(2-\vartheta \right)U\left(\vartheta \right)}\mu_{4}t\right)\right]}^{n},\\ \left\|\hbar_{5n}\left(t\right)\right\|\leq \left\|C_{En}\left(0\right)\right\|{\left[\left(2\frac{\left(1-\vartheta \right)}{\left(2-\vartheta \right)U\left(\vartheta \right)}\mu_{5}\right)+\left(2\frac{\vartheta }{\left(2-\vartheta \right)U\left(\vartheta \right)}\mu_{5}t\right)\right]}^{n}. \end{array}$$

As a result, the existence of solutions of the breast cancer model and its continuity are achieved. In addition to this, we will show that that the above is a solution of system (4) and proceed as follows:

(41) $$\begin{array}{c} C_{A}\left(t\right)-C_{A}\left(0\right)=C_{\text{An}}\left(t\right)-M1_{n}\left(t\right),\\ C_{B}\left(t\right)-C_{B}\left(0\right)=C_{\text{An}}\left(t\right)-M2_{n}\left(t\right),\\ C_{C}\left(t\right)-C_{C}\left(0\right)=C_{Cn}\left(t\right)-M3_{n}\left(t\right),\\ C_{D}\left(t\right)-C_{D}\left(0\right)=C_{Dn}\left(t\right)-M4_{n}\left(t\right),\\ C_{E}\left(t\right)-C_{E}\left(0\right)=C_{En}\left(t\right)-M5_{n}\left(t\right). \end{array}$$

Thus, we have

(42) $$\begin{array}{c} \left\|H_{n}\left(t\right)\right\|=\left\|\frac{2\left(1-\vartheta \right)}{\left(2-\vartheta \right)U\left(\vartheta \right)}\left(L_{1}\left(t,C_{\text{An}}\right)-L_{1}\left(t,C_{A\left(n-1\right)}\right)\right)+\frac{2\vartheta }{\left(2-\vartheta \right)U\left(\vartheta \right)}\times \int_{0}^{t}\left(L_{1}\left(y,C_{\text{An}}\right)-L_{1}\left(y,C_{A\left(n-1\right)}\right)\right)dy\right\|,\leq \frac{2\left(1-\ell \right)}{\left(2-\ell \right)U\left(\ell \right)}\left(L_{1}\left(t,{C_{A}}_{n}\right)\right.-\left(L_{1}\left(t,{C_{A}}_{\left(n-1\right)}\right)\right.+\frac{2\vartheta }{\left(2-\vartheta \right)U\left(\vartheta \right)}\times \int_{0}^{t}\left\|\left(L_{1}\left(y,C_{A}\right)-L_{1}\left(y,C_{A\left(n-1\right)}\right)\right)\right\|dy,\leq \frac{2\left(1-\vartheta \right)}{\left(2-\vartheta \right)U\left(\vartheta \right)}\mu_{1}\left\|C_{\text{An}}-C_{A\left(n-1\right)}\right\|+\frac{2\vartheta }{\left(2-\vartheta \right)U\left(\vartheta \right)}\mu_{1}\left\|C_{\text{An}}-C_{A\left(n-1\right)}\right\|t. \end{array}$$

Following the technique, we proceed as

(43) $$\begin{array}{c} \left\|M1_{n}\left(t\right)\right\|\leq {\left(\frac{2\left(1-\vartheta \right)}{\left(2-\vartheta \right)U\left(\vartheta \right)}+\frac{2\vartheta }{\left(2-\vartheta \right)U\left(\vartheta \right)}t\right)}^{n+1}\mu_{1}^{n+1}a. \end{array}$$

Then, the following is obtained at *t*_0_:

(44) $$\begin{array}{c} \left\|M1_{n}\left(t\right)\right\|\leq {\left(\frac{2\left(1-\vartheta \right)}{\left(2-\vartheta \right)U\left(\vartheta \right)}+\frac{2\vartheta }{\left(2-\vartheta \right)U\left(\ell \right)}t_{0}\right)}^{n+1}\mu_{1}^{n+1}a. \end{array}$$

Eq. (44) implies that

(45) $$\begin{array}{c} \left\|M1_{n}\left(t\right)\right\|⟶0,n⟶\infty . \end{array}$$

Following the same procedure, we obtain that *ℳ*2_*n*_(*t*), *ℳ*3_*n*_(*t*), *ℳ*4_*n*_(*t*), and *ℳ*5_*n*_(*t*) approaches to 0 as *n* tends to ∞.

In the next step, we focus on the uniqueness of the solution of system (4); on contrast, we assume that (*𝒞*_*A*1_(*t*), *𝒞*_*B*1_(*t*), *𝒞*_*C*1_(*t*), *𝒞*_*A*1_(*t*)) is another solution of system (4); then, we have

(46) $$\begin{array}{c} C_{A}\left(t\right)-C_{A1}\left(t\right)=\frac{2\left(1-\vartheta \right)}{\left(2-\vartheta \right)U\left(\vartheta \right)}\left(L_{1}\left(t,C_{A}\right)-L_{1}\left(t,C_{A1}\right)\right)+\frac{2\vartheta }{\left(2-\vartheta \right)U\left(\vartheta \right)}\times \int_{0}^{t}\left(L_{1}\left(y,C_{A}\right)-L_{1}\left(y,C_{A1}\right)\right)\;dy. \end{array}$$

Applying the properties of norm, the above (46) converted into the following:

(47) $$\begin{array}{c} \left\|C_{A}\left(t\right)-C_{A1}\left(t\right)\right\|\leq \frac{2\left(1-\vartheta \right)}{\left(2-\vartheta \right)U\left(\vartheta \right)}\left\|L_{1}\left(t,C_{A}\right)-L_{1}\left(t,C_{A1}\right)\right\|+\frac{2\vartheta }{\left(2-\vartheta \right)U\left(\vartheta \right)}\times \int_{0}^{t}\left\|L_{1}\left(y,C_{A}\right)-L_{1}\left(y,C_{A1}\right)\right\|dy. \end{array}$$

Here, Lipschitz condition of kernel gives the following:

(48) $$\begin{array}{c} \left\|C_{A}\left(t\right)-C_{A1}\left(t\right)\right\|\leq \frac{2\left(1-\vartheta \right)}{\left(2-\vartheta \right)U\left(\vartheta \right)}\mu_{1}\left\|C_{A}\left(t\right)-C_{A1}\left(t\right)\right\|+\frac{2\vartheta }{\left(2-\vartheta \right)U\left(\vartheta \right)}\times \int_{0}^{t}\mu_{1}t\left\|C_{A}\left(t\right)-C_{A1}\left(t\right)\right\|dy, \end{array}$$

which gives

(49) $$\begin{array}{c} \left\|C_{A}\left(t\right)-C_{A1}\left(t\right)\right\|\left(1-\frac{2\left(1-\vartheta \right)}{\left(2-\vartheta \right)U\left(\vartheta \right)}\mu_{1}-\frac{2\vartheta }{\left(2-\vartheta \right)U\left(\vartheta \right)}\mu_{1}t\right)\leq 0. \end{array}$$

**Theorem 4 .**

There exists a unique solution of breast cancer system (4) if

(50) $$\begin{array}{c} \left(1-\frac{2\left(1-\vartheta \right)}{\left(2-\vartheta \right)U\left(\vartheta \right)}\mu_{1}-\frac{2\vartheta }{\left(2-\vartheta \right)U\left(\vartheta \right)}\mu_{1}t\right)>0. \end{array}$$

**Proof**

For the required result, we assume that the above condition (50) holds true; then, (49) implies that

(51) $$\begin{array}{c} \left\|C_{A}\left(t\right)-C_{A1}\left(t\right)\right\|=0. \end{array}$$

As a result of this, we have the following:

(52) $$\begin{array}{c} C_{A}\left(t\right)=C_{A1}\left(t\right). \end{array}$$

Following similar steps, we attain

(53) $$\begin{array}{c} C_{B}\left(t\right)={C_{B}}_{1}\left(t\right),C_{C}\left(t\right)={C_{C}}_{1}\left(t\right),\\ C_{D}\left(t\right)={C_{D}}_{1}\left(t\right),C_{E}\left(t\right)={C_{E}}_{1}\left(t\right). \end{array}$$

## 4. Simulations and Discussions

In this section of the article, we perform several simulations to examine the complex dynamics of our proposed breast cancer model with adverse reaction of chemotherapy treatment at population level of patients in a hospital through the Adams-Bashforth two-step method [?]. These simulations are important in order to identify the most significant input parameters that highly disturb the population level of cancer patients. The dynamical behaviour of the fractional breast cancer system is investigated numerically to provide more accurate picture of breast cancer chemotherapy patients. The values of parameters are assumed for simulation purposes in numerical analysis of the system.

Here, we perform seven simulations to conceptualize the effect of the input parameters on the dynamical behaviour of the system. Figures 3 and 4 illustrate the dynamics of breast cancer with the variation of fractional-order *ϑ*. We observed that the index of memory *ϑ* has significant influence on the solution pathway of breast cancer model and the control of *ϑ* can highly control the dynamics of breast cancer in all the subgroups. The solution pathway of the proposed fractional-order model (4) of breast cancer with the variation of input parameter *δ*_*AD*_ is shown in Figure 5. We noticed in the second scenario that the increase of parameter *δ*_*AD*_ decreases the level of *𝒞*_*A*_ and *𝒞*_*B*_ while increases the level of *𝒞*_*C*_, *𝒞*_*D*_, and *𝒞*_*E*_. In this case, the increase of the level of subgroups *𝒞*_*C*_ and *𝒞*_*E*_ is critical in the sense to increase the cancer-induced and cardiac death rates in the patients. In the third scenario presented in Figure 6, we illustrate the dynamical behaviour of our proposed fractional-order model (4) of breast cancer with the variation of input parameter *δ*_*BD*_. It is clear that the increase of this parameter *δ*_*BD*_ will decrease the number of patients *𝒞*_*B*_ and will increase the number of patients in the subgroup *𝒞*_*D*_ which is effective. However, the population level of *𝒞*_*B*_ and *𝒞*_*E*_ increases slightly. In Figure 7, we represent the solution pathway of the fractional-order model (4) with the variation of input parameter *δ*_*BE*_. We observed that the increase of this parameter decreases the level of cancer patients in *𝒞*_*B*_ and *𝒞*_*C*_ which implies that the death rate of cancer will be decreased. However, the increase of *δ*_*BE*_ increases the level of patients in *𝒞*_*E*_, and as a result, the cardiac death rate will be increased. We perform numerical comparison of ordinary model (1) and fractional model (4) in Figure 8 with fractional order 0.9 which illustrate that fractional results are better than the ordinary one in the sense to decrease the level of different cancer stages.

In the fifth scenario presented in Figure 9, we demonstrate the time series of breast cancer model with the variation of input parameter *δ*_*CD*_. It is noticed that the increase of *δ*_*CD*_ increases the cardiac death rate while decreases the cancer death rate. In Figures 10 and 11, we visualize the solution pathway of fractional-order breast cancer model with the variation of *δ*_*CE*_ and *δ*_*DE*_, respectively. We observed that similar to the fifth scenario, the level of cancer patient decreases which leads to a decrease in the cancer death rate, while the level of cardiotoxic patient increases which increase cardiac death rate. The roles of parameters are visualized through these simulations, and one can easily understand how to lower cancer and cardiac death rate in the hospital of cancer patient. Furthermore, we observed that the control of fractional order can control the number of cancer patients, and as a result, the cancer and cardiac death rate will be controlled. Therefore, the index of memory *ϑ* is suggested to the policy makers and medical experts for the control of cancer and cardiac death.

## 5. Conclusion

It is eminent that the treatment and vaccination play a vital contribution to overcome the infectious diseases. However, sometimes the treatment and vaccination are not fully fruitful and have adverse reactions on the patient. Chemotherapy treatment is the most common treatment for breast cancer where the use of drugs affects the heart of a patient which leads to cardiotoxicity. In this article, we formulated a mathematical model for breast cancer with chemotherapy treatment at population level of patients in fractional framework to investigate the adverse reaction of chemotherapy on the heart of a patient. The proposed fractional model of breast cancer is then investigated for the basic properties through fractional calculus. The existence and uniqueness of the proposed breast cancer system are investigated through fixed point theory. Moreover, we highlighted the dynamical behaviour of our fractional system of breast cancer with the help of the Adams-Bashforth method. We have shown the dynamical behaviour of different stages of breast cancer model with variation of fractional-order *ϑ*. Our findings suggest that the index of memory *ϑ* is an important input parameter and recommended to the policy makers. Finally, the dynamical behaviour of different stages of breast cancer is highlighted numerically to show the influence of several input parameters on the time series of breast cancer. The impact of input parameters of the breast cancer system has been illustrated the most critical factors highlighted for the control and prevention of breast cancer. In future study, we will extend our model using delay differential equations to investigate the significance of time delay in breast cancer dynamics. We will also incorporate some control measures to lessen the progression of breast cancer to different stages in our future work.

## Figures and Tables

**Figure 1:** Illustration of milk making (lobules) and shuttling (ducts) glandular epithelial cells anchored by connective tissue.

**Figure 2:** Effect of anthracyclines on the heart of a patient during cancer chemotherapy.

**Figure 3:** Time series of our proposed fractional-order model (4) of breast cancer with the variation of fractional-order *ϑ*, i.e., *ϑ* = 0.6,0.8,1.

**Figure 4:** Time series of our proposed fractional-order model (4) of breast cancer with the variation of fractional-order *ϑ*, i.e., *ϑ* = 0.4,0.5,0.7.

**Figure 5:** Illustration of dynamical behaviour of our proposed fractional-order model (4) of breast cancer with the variation of input parameter *δ*_*AD*_, i.e., *δ*_*AD*_ = 0.0351,0.0651,0.0951.

**Figure 6:** Illustration of dynamical behaviour of our proposed fractional-order model (4) of breast cancer with the variation of input parameter *δ*_*BD*_, i.e., *δ*_*BD*_ = 0.242,0.442,0.642.

**Figure 7:** Time series of our proposed fractional-order model (4) of breast cancer with the variation of fractional-order *δ*_*BE*_, i.e., *δ*_*BE*_ = 0.531,0.631,0.731.

**Figure 8:** Competitive analysis of ordinary model and fractional model where the curve of blue dots illustrates ordinary model while the curve of red dots illustrates the fractional model of breast cancer.

**Figure 9:** Illustration of dynamical behaviour of our proposed fractional-order model (4) of breast cancer with the variation of input parameter *δ*_*CD*_, i.e., *δ*_*CD*_ = 0.358,0.458,0.558.

**Figure 10:** Time series of our proposed fractional-order model (4) of breast cancer with the variation of fractional-order *δ*_*CE*_, i.e., *δ*_*CE*_ = 0.296,0.396,0.496.

**Figure 11:** Time series of our proposed fractional-order model (4) of breast cancer with the variation of fractional-order *δ*_*DE*_, i.e., *δ*_*DE*_ = 0.311,0.422,0.533.

## Data Availability

The data that support the findings of this study are available from the corresponding author upon reasonable request.

## References

[1] Fitzmaurice C., Dicker D., Pain A. (2015). The global burden of cancer 2013. *JAMA Oncology*.

[2] Vasiliadis I., Kolovou G., Mikhailidis D. P. (2014). *Cardiotoxicity and cancer therapy*. *Angiology*.

[3] Mercurio V., Pirozzi F., Lazzarini E. (2016). Models of heart failure based on the cardiotoxicity of anticancer drugs. *Journal of Cardiac Failure*.

[4] Hategekimana F., Saha S., Chaturvedi A. (2017). Dynamics of amoebiasis transmission: stability and sensitivity analysis. *Mathematics*.

[5] Elaiw A. M., Elnahary E. K. (2019). Analysis of general humoral immunity HIV dynamics model with HAART and distributed delays. *Mathematics*.

[6] Byrne H. M. (2010). Dissecting cancer through mathematics: from the cell to the animal model. *Nature Reviews Cancer*.

[7] Armitage P., Doll R. (1954). The age distribution of cancer and a multi-stage theory of carcinogenesis. *British Journal of Cancer*.

[8] Alarcon T., Byrne H. M., Maini P. K. (2004). Towards whole-organ modelling of tumour growth. *Progress in Biophysics and Molecular Biology*.

[9] Dixit D. S., Kumar D., Kumar S., Johri R. (2012). A mathematical model of chemotherapy for tumor treatment. *Advances in Applied Mathematical Biosciences*.

[10] Schattler H., Ledzewicz U., Amini B. (2016). Dynamical properties of a minimally parameterized mathematical model for metronomic chemotherapy. *Journal of Mathematical Biology*.

[11] Jordao G., Tavares J. N. (2017). Mathematical models in cancer therapy. *Bio Systems*.

[12] Khajanchi S., Nieto J. J. (2019). Mathematical modeling of tumor-immune competitive system, considering the role of time delay. *Applied Mathematics and Computation*.

[13] Mahlbacher G. E., Reihmer K. C., Frieboes H. B. (2019). Mathematical modeling of tumor-immune cell interactions. *Journal of Theoretical Biology*.

[14] Enderling H., Chaplain M. A., Anderson A. R., Vaidya J. S. (2007). A mathematical model of breast cancer development, local treatment and recurrence. *Journal of Theoretical Biology*.

[15] Zhang X., Fang Y., Zhao Y., Zheng W. (2014). Mathematical modeling the pathway of human breast cancer. *Mathematical Biosciences*.

[16] Liu Z., Yang C. (2016). A mathematical model of cancer treatment by radiotherapy followed by chemotherapy. *Mathematics and Computers in Simulation*.

[17] Simmons A., Burrage P. M., Nicolau D. V., Lakhani S. R., Burrage K. (2017). Environmental factors in breast cancer invasion: a mathematical modelling review. *Pathology*.

[18] Podlubny I. (1998). *Fractional Differential Equations: An Introduction to Fractional Derivatives, Fractional Differential Equations, to Methods of Their Solution and Some of Their Applications*.

[19] Samko S. G., Kilbas A. A., Marichev O. I. (1993). *Fractional Integrals and Derivatives*.

[20] Jan R., Khan M. A., Kumam P., Thounthong P. (2019). Modeling the transmission of dengue infection through fractional derivatives. *Chaos, Solitons & Fractals*.

[21] Abdulhameed M., Vieru D., Roslan R. (2017). Magnetohydrodynamic electroosmotic flow of Maxwell fluids with Caputo-Fabrizio derivatives through circular tubes. *Computers & Mathematics with Applications*.

[22] Ucar E., Özdemir N., Altun E. (2019). Fractional order model of immune cells influenced by cancer cells. *Mathematical Modelling of Natural Phenomena*.

[23] Goufo E. D. (2015). A biomathematical view on the fractional dynamics of cellulose degradation. *Fractional Calculus and Applied Analysis*.

[24] Caputo M., Fabrizio M. (2021). On the singular kernels for fractional derivatives. Some applications to partial differential equations. *Progress in Fractional Differentiation and Applications*.

[25] Losada J., Nieto J. J. (2021). Fractional integral associated to fractional derivatives with nonsingular kernels. *Progress in Fractional Differentiation and Applications*.

[26] Dokuyucu M. A., Celik E., Bulut H., Baskonus H. M. (2018). Cancer treatment model with the Caputo-Fabrizio fractional derivative. *The European Physical Journal Plus*.

[27] El-Dessoky M. M., Khan M. A. (2021). Application of Caputo-Fabrizio derivative to a cancer model with unknown parameters. *Discrete & Continuous Dynamical Systems-S*.

[28] Caputo M., Fabrizio M. (2016). A new definition of fractional derivative without singular kernel. *Progress in Fractional Differentiation and Applications*.

[29] Losada J., Nieto J. J. (2015). Properties of a new fractional derivative without singular kernel. *Progress in Fractional Differentiation and Applications*.

